The article "Unleashing the behavioral factors affecting the decision making of Chinese investors in stock markets" was retracted in 2024. Reasons: compromised peer review; unreliable data; unreliable results or conclusions; concerns about the data.

# Unleashing the behavioral factors affecting the decision making of Chinese investors in stock markets

**DOI:** 10.1371/journal.pone.0298797

**Published:** 2024-02-13

**Authors:** Yuzhu Xia, Ghulam Rasool Madni

**Affiliations:** 1 Business School, University of Southampton, Southampton, United Kingdom; 2 Division of Management and Administrative Science, Department of Economics, University of Education, Lahore, Pakistan; Politecnico di Milano, ITALY

## Abstract

This research paper delves into the behavioral factors that have impact on decision making of Chinese investors in stock markets. As one of the world’s most dynamic and rapidly evolving financial landscapes, stock markets of China have witnessed significant growth and transformation in recent years. However, the role of behavioral biases in shaping investment decisions remains a relatively understudied aspect. Drawing upon a detailed review of studies, psychological theories, and empirical studies, this research explores various behavioral factors affecting the decision of investors at Beijing, Shanghai and Shenzhen stock markets. Through a structured questionnaire and by collecting a sample of 521 respondents, this paper investigates that herding, overconfidence, prospect, market, gamble’s fallacy, and anchoring-ability bias often lead investors to deviate from rational decision-making and contribute to market inefficiencies. While herding, prospect, and heuristic affect the investment performance in stock markets of China. Moreover, the research underscores the need for investor education programs and regulatory interventions that acknowledge the presence of behavioral biases and encourage more informed decision-making. By shedding light on these dynamics, it provides valuable insights for policymakers, financial institutions, and investors seeking to navigate the intricacies of this rapidly growing financial landscape.

## 1. Introduction

Finance pertains to the administration of funds, possessions, debts, and investments by individuals, companies, governments, and other entities. It encompasses a broad spectrum of tasks linked to the distribution, procurement, and utilization of monetary assets with the aim of accomplishing diverse objectives [1]. Finance constitutes a pivotal element in both individual and corporate spheres, aiding people and entities in making knowledgeable choices concerning the adept handling and expansion of their economic assets. Similarly, behavioral finance stands as an area of research that melds psychological principles with conventional financial theory, aiming to grasp how emotional and psychological factors impact decision-making within financial markets [2]. It acknowledges that individuals and participants in the market frequently do not solely make rational decisions when dealing with financial management and investment selections [3]. In contrast to conventional financial theories that posit participants in the market consistently make reasonable and optimal choices, behavioral finance acknowledges that human conduct frequently diverges from rationality due to psychological elements, feelings, and cognitive restrictions. Despite the multitude of theories offered by economics and finance over time, these disciplines were unable to account for instances when individuals make irrational financial judgments. Individuals are drawn to stocks due to their potential for “long-term capital growth, dividends, and as a safeguard against the erosive impact of inflation on purchasing power” [4].

While Chinese stock markets have experienced substantial growth in terms of the quantity of listed stocks and transaction values, the volatility in price trends appears to be unpredictable across various timeframes. Moreover, there exists a restricted comprehension of the behaviors exhibited by individual investors and the behavioral components that influence their choices in investment [5]. Investor decision-making is significantly influenced by behavioral aspects, which include psychological components like emotions and cognition [6].

Numerous theories [7–9] assume that investors respond rationally by thoroughly evaluating all accessible information prior to making investment choices. Some other studies [10–12] have indicated that the rationality assumption does not align with reality. It is highlighted that investors do not conform to the rational suppositions of conventional finance theories. It has been emphasized that investors do not function as “calculative utility maximizing machines,” as postulated by conventional finance theories [12]. In greater detail, individuals are susceptible to their emotions and sentiments, often leading to cognitive errors [13]. To make more precise forecasts and decisions for endeavors of investors, it is crucial to delve into the behavioral variables impacting individual investors’ decision-making processes. Behavioral finance, grounded in psychology, proves advantageous in this context, as it elucidates the reasons behind individuals’ stock purchases or sales [6].

Many scholars believe that using behavioral finance as a framework will help them to better understand that how emotion and cognitive biases affect how they make financial decisions [14]. Advocates of behavioral finance claim that by including social sciences like psychology, it is possible to understand how the stock market behaves and how market bubbles and crashes occur [15]. The significance and appeal of applying behavioral finance to the Chinese stock markets stem from two key reasons. Firstly, behavioral finance remains a relatively novel area of study. It is only recently that it has been acknowledged as a viable model for elucidating the decision-making processes of financial market investors and their subsequent influence on financial markets themselves [16]. Secondly, Asian investors in particular have been found to be more prone to cognitive biases than people from other cultural backgrounds, according to a combination of subjective, academic, and experimental findings [16]. As a result, behavioral considerations must be considered when examining the variables that influence Chinese investors’ decision-making processes.

Behavioral finance investigations have predominantly been conducted within the developed economies of USA and Europe [17]. However, compared to their use in industrialized markets, behavioral finance ideas have been applied far less frequently in developing economies. The goal of this paper is to understand the motivations behind the actions taken by investors in Chinese stock markets via the lens of behavioral finance. The pursuit of comprehending and adequately explaining investor decisions necessitates an exploration into the behavioral factors influencing these decisions within the context of the Chinese stock markets, as well as an examination of the resultant impacts on investment performance [18].

This study, which departs from earlier research that was mostly based on conventional financial theories, applies behavioral finance principles. Moreover, while preceding research has often limited its focus to specific dimension of behavioral factor [19], this research adopts a more comprehensive array of behavioral determinants in evaluating their impact on Chinese investors. Furthermore, this study expands the application of principles of behavioral finance in context of emerging stock markets of China. Additionally, the methodology employed for gauging investment performance in this research diverges from past approaches that drew on secondary data from investors’ outcomes in the securities markets. Instead, this study directly engages individual investors by asking them to assess their own success in light of factors like investment return rate and fulfilment levels. These findings extend beyond individual investors, proving useful for security organizations as a reference point for market trend analysis and prediction.

## 2. Earlier literature and hypothesis

The Efficient Markets Hypothesis (EMH) holds that markets are rational. Additionally, the theory posits that markets formulate unbiased forecasts instead of attempting to predict the future. In contrast, behavioral finance departs from this notion by asserting that financial markets can occasionally lack informational efficiency [20]. This is due to the recognition that individuals are not always guided by rationality, often making financial decisions driven by behavioral biases. When decisions deviate from rational reasoning, it becomes imperative to recognize the impact of these behavioral biases [21]. Recent investigations have delved into the consequences arising from the actions of less-than-rational agents, employing various theoretical models. Researchers have empirically tested behavioral biases [11], providing evidentiary support. However, despite the controlled environment that can be achieved through well-designed experiments [22], testing behavioral finance theories has only occasionally used a small number of experiments.

The variables related to decision-making of investors can be divided into four groups: heuristic, prospect, market, and herding. Heuristics are practical rules that help with decision-making, especially when situations are complex and uncertain [23]. Heuristics are mental shortcuts or rules of thumb that simplify decision-making. In investment, heuristics allow investors to make quick judgments based on limited information [24]. They can be beneficial as they streamline complex investment choices into manageable decisions. For Chinese investors, heuristics might help in rapidly evaluating stocks or investment opportunities in a fast-paced market environment. They make it easier to estimate probabilities and predict values by breaking them down into simpler judgments [10]. The heuristic theory includes two factors called the Gambler’s fallacy and Overconfidence [25]. The idea that a small group can represent the larger overall population it comes from is called the "law of small numbers" [12, 26], and this can lead to the Gambler’s fallacy happening [27]. In context of stock market, Gambler’s fallacy materializes when individuals inaccurately anticipate reversals in trends that are perceived as the culmination of favorable (or unfavorable) market returns [6]. The five distinct heuristic components under investigation in this study are overconfidence, anchoring, availability bias, gambler’s fallacy, and representativeness. shares. Representativeness denotes the extent to which an event bears similarity to its parent population or exhibits resemblance to that population [28]. This concept can introduce certain biases, such as the tendency for individuals to assign excessive significance to recent experiences and disregard the overall long-term average [29]. Additionally, representativeness contributes to what is referred to as “sample size neglect,” which raised when an individual attempt to infer conclusions from an insufficient number of samples [12]. Within context of stock market, application of representativeness becomes apparent when investors opt to purchase “hot” stocks as opposed to those that have performed poorly. This inclination towards representativeness offers an explanation for investor overreactions. When people overestimate dependability of their abilities and knowledge, overconfidence results [28, 30]. A range of studies [31] have indicated that excessive trading is one of the consequences observed among investors due to this phenomenon. Research offers evidence that financial analysts tend to adjust their evaluations of a company at a gradual pace, even when strong indications suggest that the initial valuation is no longer correct [32]. Overconfidence is posited to enhance traits such as persistence, mental agility, and risk broad-mindedness. Essentially, it can contribute to strengthening professional enactment. It’s worth noting that overconfidence can also influence how others perceive an individual’s capabilities, potentially expediting promotions and extending investment horizons [33].

Prospect theory elucidates the theoretical relationship between prospects and investment decisions. The theory posits that individuals make decisions based on potential gains and losses relative to a reference point, rather than focusing solely on final outcomes [34]. Prospect theory suggests that individuals perceive outcomes relative to a reference point, often the status quo or an initial investment value. Investors evaluate gains and losses based on this reference point [35]. It is also highlighted by the theory that losses loom larger than equivalent gains. Investors tend to exhibit loss aversion, being more sensitive to potential losses than to gains of equal magnitude. This asymmetry significantly influences investment decisions, leading to risk-averse behavior to avoid potential losses [22]. Prospect theory shapes risk preferences in investment choices. When faced with potential gains, individuals might exhibit risk-seeking behavior, willing to take chances for further gains. Conversely, when facing potential losses, they tend to become risk-averse, prioritizing capital preservation over potential gains [18]. Understanding prospect theory aids in comprehending how investors evaluate investment opportunities, perceive risks, and make decisions based on potential gains and losses. The asymmetrical impact of gains and losses, reference points, and framing effects significantly shape investment choices, risk preferences, and the overall decision-making process in financial markets [36].

Efficient Market Hypothesis (EMH) suggests that markets efficiently incorporate all available information, making it challenging to outperform the market consistently. Under this theory, investors believe that attempting to beat the market through individual security selection or timing is futile, leading to passive investment strategies like index funds [13]. Behavioral finance challenges the EMH by highlighting investor behavior that deviates from rationality, leading to market anomalies [21]. Psychological biases, herding behavior, overreaction, and under reaction to news or market events can cause price distortions or inefficiencies. Investors identifying these anomalies might capitalize on mispriced assets, impacting their investment decisions. Market sentiment, driven by collective investor emotions, influences investment decisions [32]. Positive sentiment might lead to increased buying and inflated asset prices, while negative sentiment can trigger selling pressure and price declines. Investors might adjust their portfolios based on market sentiment, impacting their decisions [9]. The degree of market efficiency influences investors’ choice of investment strategies. In highly efficient markets, investors might opt for passive strategies, while in less efficient markets, active strategies that attempt to exploit mispriced assets might be preferred [37]. The market significantly influences investors’ perceptions of risk and return. In bull markets with rising asset prices, investors might perceive lower risk and higher potential returns, leading to more aggressive investment decisions [26]. Understanding the relationship between the market and investment decisions involves considering market efficiency, behavioral biases, sentiment, analysis methods, and the interplay between risk and return perceptions. These factors collectively shape how investors interpret market information and make investment decisions within financial markets [38].

The relationship between herding behavior and investment decisions is rooted in the influence of social dynamics on investor behavior within financial markets. Herding refers to individuals imitating the actions of a larger group rather than making independent decisions. In investment contexts, herding occurs when investors follow the crowd, mimicking others’ actions without conducting thorough individual analysis [25]. Herding often emerges due to information cascades, where individuals base their decisions on the actions of others rather than on private information. Initially, a few investors might make decisions based on their information or analysis. Subsequent investors observe these actions and may choose to follow suit, leading to a cascade of others mimicking these decisions, irrespective of personal information or analysis [31]. Herding behavior can lead to market inefficiencies and price distortions. When a significant number of investors herd towards certain assets, it can create artificial demand or supply, causing prices to deviate from their fundamental values [11]. This creates opportunities for contrarian investors who recognize the herd’s influence and trade against prevailing market sentiment [23]. Herding behavior can significantly influence investment decisions. Fear of missing out (FOMO) or assuming safety in numbers might drive investors to join the herd. Conversely, some investors might be contrarians, leveraging opportunities created by herd-driven mispricing [39]. Acknowledging the impact of herding behavior helps investors navigate market trends and potentially capitalize on opportunities arising from herd-driven mispricing [40]. In light of above discussion, hypothesis *H1* is put forth as follows:

***H1*:** *The behavioral elements such as heuristics*, *prospect*, *market*, *and herding have positive influence on investment decisions of Chinese investors*.

Behavioral factors can positively influence the investment performance of Chinese investors through several theoretical perspectives. Behavioral finance theory suggests that market inefficiencies arise due to investors’ behavioral biases. These biases, such as overreaction to news, herding behavior, or cognitive errors, create opportunities for skilled investors to exploit mispricing [23]. Behavioral biases might lead to certain stocks being undervalued or overvalued, allowing astute investors to identify mispriced assets and capitalize on them, ultimately enhancing investment performance [12]. Adaptive Market Hypothesis posits that markets continuously adapt to the behavior of investors. Investors’ behavioral tendencies, such as herd behavior or biases in risk perception, might contribute to temporary price distortions [34]. However, over time, market mechanisms adjust, and prices reflect fundamental values. Skilled investors who recognize and navigate these behavioral fluctuations can outperform the market by exploiting short-term misalignments before market corrections occur [26, 41]. Traditional portfolio theory assumes rational, utility-maximizing investors. However, behavioral portfolio theory acknowledges investors’ behavioral biases and their influence on portfolio construction. Investors might exhibit biases like home country bias (overweighting domestic assets) or familiarity bias (preferring familiar stocks), which might lead to portfolios deviating from efficient diversification [35]. However, if investors understand and manage these biases effectively, they can construct portfolios that capitalize on market opportunities and enhance performance. Prospect theory suggests that investors’ risk attitudes differ when facing gains or losses [18]. Understanding how investors perceive gains and losses can lead to better risk management strategies. Investors might adopt strategies that focus on capital preservation when facing potential losses and pursue more aggressive strategies to capitalize on gains. Effectively managing risk based on these behavioral tendencies can positively impact investment performance [33]. In summary, behavioral factors can positively influence investment performance by providing opportunities to exploit market inefficiencies, adapt to behavioral fluctuations, construct portfolios aligned with behavioral biases, and employ effective risk management strategies based on investors’ perceptions of gains and losses. Understanding these behavioral aspects enables investors to navigate the market more strategically, potentially leading to improved investment outcomes.

In their research [34], Lin and Swanson examined investment performance using five different time spans and three measures of returns. The study found that investors can attain higher returns, especially in the short run. This increased performance isn’t necessarily due to taking on more risk, but rather is connected to short-term price trends [42]. However, when compared to performance over longer periods, this impressive performance becomes weaker or declines. This suggests that short-term factors like a higher demand for previously successful stocks and/or an oversupply of stocks that have performed poorly in the past contribute to achieving outstanding enactment. In short run, but not over long time periods, behaviors have the effect of pushing up equities with a history of high performance and pushing down stocks with a history of negative performance [36]. The predominance of short run performance, especially when powered by the momentum of winners rather than losers, suggests that buying behavior adds fresh knowledge to market.

The study conducted by [35] explores the degree of impact that overconfidence exerts on investment performance, as measured by two primary indicators: investment return rate and swapping experience. The investment coming back rate, or profit, serves as an objective measure of investment performance, gauged by investors in relation to the profit rates achieved by their peers [43]. On the other hand, an investor’s trading experience signifies the duration for which an individual has been participating in securities markets. The finding of research show that while overconfidence does not significantly influence investment profit, it does exert an impact on the trading practice of separable investors [12, 28–31].

In conclusion, there exists a plethora of methods for evaluating stock investment performance. Previous researchers have predominantly relied on secondary data gathered from investors’ activities in the securities markets to gauge investment performance [16, 34]. In order to go deeper, the return on stock investments is evaluated using both objective and subjective criteria. Comparing actual return degrees to the normal return rate of the securities market is what is required for impartial assessment [25]. Furthermore, this study adds another factor to evaluate investment performance: level of satisfaction with investment decisions. In real-world scenarios, certain investors might be pleased with their investment performance even profits aren’t significant, whereas others might be dissatisfied despite having relatively high profits [18]. Based on the discussions provided, it’s logical to suggest that behavioral factors have an impact on the investment choices. This idea forms the basis for creation of hypothesis *H3*:

***H2*:** *Behavioral factors have positive influence on investment performance of Chinese investors*.

## 3. Materials and methods

### 3.1. Sample and data collection

To comprehend the typical behaviors exhibited by individual investors, a cross-sectional design is chosen as the most appropriate approach, in contrast to case studies, experiments, or longitudinal-designs [13]. Specifically, experimental designs often prove effective for investigating the relationships between variables. Among the array of data collecting approaches available, the self-completion method is selected for gathering quantitative data. Self-completed questionnaires are widely employed in quantitative research due to their convenience for respondents, particularly when sensitive information is involved [36]. The convenient sampling method is adopted to collect the data to ensure representation across various demographics because it is best way to get the highest response rate and saving the money and time. It is worth noting that convenience sampling is a type of non-probability sampling and its results cannot be generalized [37]. Questionnaires are distributed to investors via email and social media platforms. Regarding geographical distribution, the respondents were sourced from various regions across China, contributing to a broader representation within the study. The questionnaires were sent to individual investors randomly through brokers of security companies registered in Beijing, Shanghai and Shenzhen stock markets of China. The investors from ten leading securities companies have been selected. The survey was carried out from February 1, 2023 to May 30, 2023. The “Ethical Committee” of University of Education approved the study. A written consent was gained from participants of the study. A total of 700 questionnaires are disseminated to investors to facilitate the research objectives. There are three parts of questionnaire including personal details, behavioral factors affecting investment choices, and investment performance. A set of questions has been developed to encompass all aspects described in theories of behavioral finance. Within these parts, we’ve utilized a 6-point Likert scale, a commonly employed technique for collecting opinions and attitudes from participants [38, 39]. Individual investors are requested to express their consent to express the impact of behavioral factors on their investment decisions and their alignment with statements related to investment performance. The scale covers a range from 1 to 6, encompassing options such as "strongly disagree," "disagree," "somewhat disagree," "somewhat agree," "agree," and "strongly agree." To ensure the soundness of opinion poll, draft is tested by experts in the field as well as by fifty individual investors. Subsequent to these iterations, the final version of the questionnaire is prepared.

The data acquired from the questionnaires offer foundational insights into the factors that influence investors’ decisions. Given the research’s focus on exploring behavioral factors, it’s advisable to employ a comparatively large sample size. A larger sample size enhances representativeness and consequently bolsters the reliability of the findings [37]. According to [38], for quantitative research, a minimum of 100 respondents is recommended to ensure compatibility with statistical methods of data analysis.

### 3.2. Methodology

The gathered data is subjected to processing and analysis through the utilization of SPSS and AMOS software. The initial step involves data cleaning, where questionnaires showing poor quality, such as excessive misplaced values or biased ratings, are excluded from the dataset. Subsequently, a range of statistical methods is employed to meet the research objectives. Descriptive statistics, factor analysis, the Cronbach’s Alpha test, and structural equation modelling (SEM) are among the used approaches.

The exploratory factor analysis (EFA) in this study employs several criteria, including Factor Loadings, Kaiser-Meyer Olkin Measure of Sampling Adequacy (KMO), Total Variance Explained, and Eigenvalue. When factor loadings are above 0.5, it indicates practical significance in EFA [38]. A KMO score in range of 0.5–1.0 (with a significance level below 0.005) confirms the appropriateness of factor analysis for the data [40]. The study uses Cronbach’s Alpha Test to assess reliability of variables [41]. According to Nunnally’s suggestion [42], the value of Cronbach’s alpha of 0.7 is considered to indicate measurement reliability. However, some statisticians consider an alpha value higher than 0.6 to be acceptable [43].

SEM is utilized to validate how behavioral factors influence investment performance of individual investor. Additionally, it’s used to estimate the strength of relationships among these factors. The model is considered satisfactory if it meets the following criteria: “a squared error of approximation (RMSEA) equal to or less than 0.10, a comparative fit index (CFI) equal to or greater than 0.90, and a parsimonious fit index (PFI) equal to or greater than 0.60” [44].

Respondents are provided with comprehensive and pertinent information to enable them to willingly participate in the research. Each questionnaire includes a cover page that furnishes adequate details about the study, thereby allowing respondents to make informed decisions regarding their participation. Furthermore, the distribution of questionnaires occurs through email and social media platforms, granting respondents the autonomy to choose whether or not to respond. It’s important to emphasize that respondents were informed about the survey’s commitment to maintaining their anonymity and confidentiality throughout the process.

### 3.3. Empirical findings

Out of the 700 questionnaires distributed to individuals, 521 respondents have been recorded, resulting in a response rate of 80%. This rate stands as moderately high, particularly for a postal questionnaire survey. A breakdown of the respondent sample by characteristics such as gender, age, duration of participation in the stock market, total investment amount, and more, has been carried out.

The gender composition of the sample shows that female investors account for 47% of the participants, while male investors account for 53%. In terms of age distribution, 77% of stock investors (or 77% of the whole sample) are in the age of 26–35. Furthermore, 12% of respondents are in age of 36–45, while 9% are in age of 18–25. This distribution emphasizes that a significant number of individual investors are under the age of 35, indicating that this study is likely to substantially represent the investment behaviors of this age group. Regarding the age skew toward younger respondents, this might reflect a higher engagement of younger demographics in stock market participation.

An analysis of the duration of participation in the stock market reveals that 33% of respondents have been engaged for less than 3 years, 22% have participated for 3 to fewer than 5 years, 15% have been involved for less than 1 year, while 29% have taken part in the stock marketplace for over five (5) years but less than ten (10) years. A mere 1% have an extensive history of more than 10 years of participation in stock market.

Concerning investment ranges, respondents cover the spectrum from US$2000 to US$30000. Notably, the greater proportions of individual stockholders in the sample are invested within the ranges of US$2000–10000: 35% investing less than US$2000, 32% investing between US$2000–4000, and 30% investing between US$4000–10000. Moreover, a small portion of the sample, 3%, invests substantially higher amounts exceeding US$30000.

The EFA has been applied to set of communicative variables and investment in order to discern the underlying factors to which these variables pertain. Through several iterations involving the removal of unsuitable variables, the remaining variables have been successfully grouped into six distinct factors. These factors consist of five factors associated with communicative variables and one factor linked to investment performance. The decision to stop at an Eigenvalue of 1.00 has been made, resulting in a Kaiser-Meyer Olkin (KMO) measure of 0.77 (with a significance level of 0.000). This measure, along with a percentage of total variance explained at 71.41%, validates the suitability and acceptance of the factor analysis for these variables. Moreover, all factor loadings have exceeded the threshold of 0.5. The combination of these indices serves as conclusive evidence supporting the appropriateness of conducting factor analysis on these variables. Further details and findings are outlined in Table 1.

**Table 1:** Factor analysis.

Factor	Variables	Factor Loading	Cronbach’s Alpha	CR	AVE	F Test
Herding	1. The investment choices made by other investors influence your own decisions regarding the types of stocks to choose.	0.88	0.91	0.85	0.71	25 (0.00)
	2. The choices of other investors concerning the capacity of stocks they choose to invest in affect your own investment decisions.	0.84				
	3. The investment choices of other investors, both purchasing and marketing stocks, influence your own decisions regarding investments.	0.86				
	4. You tend to respond promptly to shifts in the decisions of other investors and align your actions with their response in stock market.	0.80				
Prospect	5. Following a previous loss, you tend to become more cautious and risk-averse in your approach.	0.82	0.88	0.88	0.74	35 (0.01)
	6. You prefer to avoid selling shares that have declined while being more likely to sell shares that have increased in value.	0.80				
	7. You typically manage each component of your investment portfolio as separate entities.	0.79				
	8. You disregard the interconnections among various investment opportunities.	0.80				
Market	9. You meticulously evaluate the price fluctuations of stocks you are considering for investment.	0.83	0.89	0.89	0.70	4 (0.03)
	10. Market information holds significance in your stock investment decisions.	0.84				
	11. You take into account the historical trends of stocks you are contemplating for investment.	0.81				
Overconfidence and Gambler’s fallacy	12. You are convinced that your knowledge and comprehension of the stock market will enable you to outperform the market as a whole.	0.85	0.785	0.83	0.77	45 (0.01)
	13. You typically have the ability to predict the conclusion of favorable or unfavorable outcomes.	0.82				
Anchoring and Ability bias	14. You predict alterations in future stock prices by analyzing recent stock price movements.	0.85	0.86	0.84	0.69	36 (0.00)
	15. You have a preference for investing in domestic stocks over international ones due to the greater availability of information regarding local stocks.	0.80				
Investment Performance	16. The current rate of return on your stock investment corresponds to the expected outcome.	0.90	0.92	0.89	0.79	12 (0.00)
	17. Your investment returns are on par with or better than the average market performance.	0.89				
	18. You are satisfied with your investment decision during the last year, which included selling, purchasing, stock selection, and stock quantity determination.	0.85				

RMR = 0.045 RMSEA = 0.048

CFI = 0.948 GFI = 0.925

RFI = 0.962 NFI = 0.932

IFI = 0.948 Normed chi square (x^2^ / df) = 2.993 p < 0.001

Note: RMR, IFI, RMSEA, CFI, GFI, RFI, and NFI stand for “root mean square residual, incremental fit index, root mean square error of approximation, comparative fit index, goodness of fit index, relative fit index and normed fit index” respectively.

Composite reliability (CR) and Cronbach’s α are used to assess the dependability of constructs. The values of Cronbach’s α and CR demonstrate strong internal reliability. Next, discriminant and convergent validity are evaluated. To establish convergent validity, factor loadings should be at least 0.50, and Average Variance Extracted (AVE) coefficients should also reach 0.50. The findings revealed that all items exhibited factor loadings surpassing 0.50, and AVE coefficients exceeded 0.50, indicating robust convergent validity. Several goodness of fit indices are employed to determine the adequacy of model. The ratio of (x2/df) was less than 5, and the RMR score was 0.045, with the RMSEA score at 0.048, both falling below the acceptable threshold of 0.08. Moreover, the values of GFI, CFI, RFI, NFI, and IFI all exceeded the recommended threshold of 0.90 [38]. Thus, based on these indicators, the data demonstrated a strong fit to the measurement model.

The herding, prospect, and market variables are combined into a single interconnected factor, as indicated in Table 1. Conversely, the heuristic variables are split between two factors: overconfidence-gambler’s fallacy and anchoring-ability bias. This finding slightly differs from Hypothesis H1, which suggested classifying behavioral variables into four groups. As a result, there are five main behavioral aspects that influence individual investors’ investment decisions. The Cronbach’s α test ensures the consistency of the items within these categories determined by factor analysis. This evaluation ensures the measurements’ dependability for future usage. The results reveal that the Cronbach’s α values for all factors are greater than 0.6, and the significance of the F-test for each factor is less than 0.05. These findings show that the items within the factors are reliable, making them acceptable for further investigation.

The average values of each variable in the sample are employed to gauge the extent of influence that behavioral variables have on investment decisions. Likewise, the investment performance variables are evaluated by computing the average ratings given by respondents for each variable. Since 6-point scale is used, their average value act as indicators of their effect on investment decision-making, as outlined below:

- Mean value less than 2 shows very little impact from the factors.
- Mean values ranging from 2–3 show that variables have little impact.
- Mean values ranging from 3–4 show that variables have moderate impact.
- Mean values ranging from 3–4 show that variables have significant impact.
- Mean values greater than 5 show that variables have substantial impact.

The impact of each factor is shown in the following Table 2:

**Table 2:** 

Factor	Variable	Mean	Standard Deviation
Herding	1. The investment choices made by fellow investors influence your own decisions regarding the types of stocks to select.	3.58	1.22
	2. The investment choices of other investors regarding stock volumes affect your own investment decisions.	3.53	1.43
	3. Your personal investment selections are influenced by the stock purchases and sales made by other investors.	3.18	1.22
	4. You have a propensity to react quickly to changes in other investors’ trading strategies and mimic their responses.	2.85	1.74
Prospect	5. Following a previous loss, you exhibit an increased tendency towards risk aversion.	3.52	1.54
	6. You frequently hesitate to sell shares whose value has decreased but are quick to do so when the value has increased.	3.63	1.52
	7. You have a propensity to evaluate every element of your investing portfolio separately.	4.06	1.21
	8. You fail to consider how different investing opportunities are related.	3.52	1.31
Market	9. You carefully examine the price swings of the stocks you intend to buy.	4.44	1.30
	10. Gathering market data is important for your stock investment strategy.	4.51	1.41
	11. You take into account the past trends of stocks when making investment decisions.	4.46	1.23
Overconfidence and Gambler’s fallacy	12. You hold the belief that your stock market expertise and knowledge can enable you to achieve better results than the overall market performance.	3.31	1.20
	13. You typically possess the ability to predict the conclusion of favorable or unfavorable outcomes.	2.80	1.87
Anchoring and Ability bias	14. You predict alterations in future stock prices by analyzing recent stock price movements.	3.79	1.51
	15. You have a preference for purchasing local stocks over international ones due to the greater availability of information about local stocks.	3.72	1.81
Investment Performance	16. The rate of return from your recent stock investment aligns with your anticipated outcome.	2.87	1.19
	17. As of late, your rate of return is either comparable to or higher than the industry standard.	2.57	1.53
	18. You are satisfied with investing decisions you made during last year, including buying, selling, choosing stocks, and figuring out volumes.	2.74	1.82

This study shows that the representativeness-related characteristics are not reliable enough to be taken into account as behavioral influences on the choices made by individual investors. On the other hand, overconfidence, anchoring, and ability bias have only little effects on how individual investors make decisions. Contrarily, the gambler’s fallacy has no impact on their choice of investments. All three behavioral tendencies; regret aversion, loss aversion, and mental accounting are depicted through variables in the Prospect dimension that affect investment decisions of stock investors. Individual investors exhibit a moderate level of mental accounting, regret aversion, and loss aversion. Notably, these investors demonstrate a strong inclination toward treating each element of their investment portfolio as a separate entity. This implies that individuals tend to thoroughly assess all accessible stock market information, including general data, historical price patterns, and current price changes, before finalizing investment choices. When contrasted with their average values, the relatively significant standard deviations of these variables suggest that certain investors attach substantial importance to market-related factors while making decisions about which stocks to purchase. Individual investors exhibit a moderate inclination to follow the trading decisions of their peers. However, it appears that the steering effect does not have an immediate impact on their stock investment adoptions.

Collectively, the mainstream of behavioral variables across the Heuristic, Prospect, and Herding factors exert reasonable impact on decision making of investors. A small number of items exhibit low impacts on investors’ choices. Conversely, certain variables within the Market and one variable within the Prospect factor are reported to exert significant influence on investment choices. The findings do not support second hypothesis that proposed all behavioral finance factors would strongly influence individuals’ investment decisions.

SEM, or structural equation modelling, is used to show how different variables relate to one another. SEM is a framework that combines elements of multiple regression and factor analysis. CFA, a component of SEM is used to confirm that factors and each of their individual components—which were discovered by Exploratory Factor Analysis, as was previously mentioned—are appropriate for inclusion in the overall model. The second part also includes multiple regression, which determines the correlation coefficients between behavioral factors, which serve as independent variables, and the investment performance factor, which serves as a dependent variable.

The results of SEM are presented in Fig 1. The GFI (Goodness-of-Fit Index) for the structural model stands at 0.95, the TLI (Tucker-Lewis Coefficient) at 0.96, the CFI at 0.95, the RMSEA at 0.08, the CMIN/df at 2.25, and the p-value is 0.00. These results indicate a strong fit between the model and data. These indicators highlight the model’s effectiveness in predicting the studied data accurately. The estimated weights for variables in a regression are displayed in Fig 1.

**Fig 1:** SEM for behavioral factors and investment performance. Note: Regression weights are mentioned above the arrows. https://docs.google.com/document/d/1olllsnBahvyWQj_Fo9ZItL6gw8g9TbpZ/edit?usp=sharing&ouid=104935469773789258540&rtpof=true&sd=true.

Three elements, Herding, Prospect, and Heuristic have an impact on Investment Performance. The fact that there are greater than 0.5 factor loading between each factor and its component variables supports the congruent validity of the data measures. A regression estimate of 0.71 (p 0.01) shows that the Overconfidence and Gambler’s fallacy heuristic behaviors have the greatest positive influence on investment performance. A regression estimate of 0.42 (p 0.01) shows that herding behaviors have a beneficial impact on investment performance, whereas a regression estimate of -0.25 (p 0.05) shows that prospect behaviors, such as following the herd, have a negative effect on investment success. These three sorts of actions together explain 52% of the variation in the success of individual investors.

The findings imply that enhancing both heuristic and herding behaviors while being mindful of the adverse effects of prospect behaviors could lead to an enhancement in investment performance. Surprisingly, a notable finding is that, despite the perception that market factors have a substantial impact on investing decisions, investors’ performance is not significantly impacted. The results derived from SEM contradict Hypothesis H2, which posits that all behavioral factors contribute positively to investment performance. In reality, only the herding and heuristic factors are recognized to exert favorable influences on investment performance. Conversely, the market factor lacks impact, and the prospect factor exhibits a negative impact on investment performance.

## 4. Analysis and discussion

The findings indicate a differentiation within the heuristics components, now labeled as Overconfident & Gambler’s fallacy and Anchoring & Availability bias. The results highlight that investors’ decisions are affected by the information available to them, particularly among the four heuristic factors, which have demonstrated sufficient reliability and consistency in measurement. Investors exhibit a preference for local stocks over international ones, attributed to the ease with which they can obtain information about local stocks through their social connections, like friends and relatives. This is consistent with a previous study’s findings [12, 45–47], which showed that 96% of investors examined have a home-market bias and disregard the benefits of diversifying their investment portfolios. The findings also reveal that individual investors possess a moderate level of confidence. This can be attributed to the fact that the security market is still in its emerging stages, resulting in complex and unpredictable fluctuations. These fluctuations can occur irrespective of the performance of the listed companies issuing the stocks [48].

While the Gambler’s fallacy has been established as a dependable variable influencing investors’ decision-making, its impact level remains quite low. This implies that investors typically lack the capability to foresee the outcomes of positive or negative market trends. This outcome is readily understandable given the substantial fluctuations in market trends, coupled with investors’ moderate level of confidence. Notably, this finding diverges significantly from the results of a previous study [45], which suggests that a majority of investors possess the ability to accurately anticipate stock price changes. Loss aversion, regret aversion, and mental accounting are the three significant prospect factors that notably impact investors’ decisions. Additionally, mental accounting serves as the fourth influential factor [49]. This finding affirms the tendency of investors to treat each component of their investment portfolio in isolation, effectively disregarding potential connections between different investment opportunities, as previously noted in a study [46]. However, this approach can lead to inefficiencies and inconsistencies in decision-making processes.

It is found that the herding variables’ significant observed influence on investors’ judgments is merely minimal. Herding tendencies are more prevalent in emerging markets than in established ones [37, 50], because of greater government intervention and lower-quality information disclosure [47]. It’s said that herding behaviors had a huge impact on Asian nations in 1997–1998. The stock market has been operational for more than a decade, which may account for the herding factor’s mild impact. As a result, investors might have accumulated greater knowledge and skills, allowing them to leverage diverse information sources prior to making investment decisions. Consequently, the effect of herding may have diminished over time [48, 51, 52]. Farber, et al. [53] emphasize the significant prevalence of the herding effect within Vietnam’s stock market, particularly directed toward positive market returns. Chen, et al. [54] posit that herding tendencies are more pronounced in emerging markets compared to developed ones due to higher levels of government intervention and lower quality of information disclosure. Additionally, Kaminsky and Schmukler [55] assert that during the period spanning 1997–1998, herding behaviors notably influenced the trajectories of Asian countries.

Three distinct groups of factors-herding, prospect, and heuristics-exert effects on investment performance. Heuristics and herding have favorable effects within these, whereas prospect has a detrimental impact on investing success. The heuristics factor, in particular, exerts a positive impact, implying a direct correlation between overconfidence, gambler’s fallacy, and investment outcomes. Investors tend to believe that heightened confidence leads to more resolute actions. In the realm of business, making decisive choices is crucial for capitalizing on significant opportunities [56]. Confident investors are likely to leverage their expertise and knowledge in specific situations, potentially enhancing investment outcomes. Regarding loss aversion, investors acknowledge it as a prevalent behavior among their peers; however, they recognize that it can result in poor trading decisions that negatively influence investors’ wealth. This perspective aligns with the viewpoints of previous studies [52]. The notion is that prior gains can fuel a sense of greed, pushing investors to seek even greater profits by investing more capital. Consequently, when unforeseen events occur, resulting losses tend to be considerably higher than anticipated. Conversely, experiencing a loss prompts individuals to become more risk-averse and cautious [57]. They approach decisions with a heightened sense of circumspection, seeking extensive information and analyzing it meticulously. They only commit to investments when confident of success. This viewpoint aligns with the perspective put forth by Odean [56]. Manager A suggests that following a profit, individuals often experience increased confidence in their decision-making abilities, prompting them to rush their judgments. This haste might cause them to undervalue or disregard crucial information that could impact investment outcomes. Notably, individuals in this scenario tend to prioritize their own judgments over external opinions, potentially leading them to overestimate the probability of success. The earlier research [57, 58] posit that during declining periods, market liquidity significantly diminishes. This occurs as buyers aim to purchase stocks at the lowest possible price while sellers seek to offload stocks at the highest possible price. Consequently, the process of selling underperforming stocks becomes more challenging compared to selling those that have gained value.

Numerous authors also assert the benefits of overconfidence. Choosing common stocks that outclass the market is a challenging endeavor, characterized by low predictability and noisy feedback. Consequently, stock selection stands as a task where people exhibit heightened overconfidence [24]. According to some researchers, overconfident investors trade at levels that are much greater than those of rational investors, potentially having a considerable impact on trading volume, market depth, wealth distribution, and other outcomes [29, 59]. Severe under-confidence and severe overconfidence are unlikely to continue over the long term, according to a study [49]. Moderate overconfidence, however, has the potential to outlast and rule logical behavior. Additionally, under certain conditions, overconfident traders may perform so well that they eclipse "rational" traders. These analytical findings have their origins in the psychological finding that overconfidence is a characteristic that is often present [35, 60].

Herding factor has a beneficial effect on investment performance in addition to the heuristics factor, represented by overconfidence. It has been proposed that in the securities market, overconfidence can encourage herding behaviors [50]. Herding behavior, often referred to as the “crowd effects,” occurs when individuals replicate others’ decisions and is frequently linked with significant stock price fluctuations or excessive volatility [51]. Consequently, emulating these prevailing trends might assist investors in enhancing their investment outcomes. This is especially important for investors who are not risk-takers because doing as the "crowd" suggests is a wise move to ensure at least average returns. Furthermore, herding contributes to notable increases in trading volumes [15, 61], consequently bolstering liquidity. As a result, investors stand to benefit from rapid capital turnover, translating to improved returns. However, it’s important to note that while herding investors aim to match their peers’ performance, non-herding traders strive to surpass competitors [22, 60]. Therefore, achieving higher returns necessitates careful consideration of the potential positive and negative effects of herding before making choices regarding investments [25].

However, it’s essential to acknowledge that every investment inherently carries a degree of risk, and without assuming some level of risk, high returns cannot be pursued. While careful consideration is prudent before making decisions, excessive caution might lead to delayed actions, potentially causing investors to miss out on favorable investment opportunities and subsequently reducing their prospects for achieving substantial profits [31].

## 5. Conclusions

Five key behavioral factors, including herding, market, prospect, overconfidence, and anchoring-ability bias, influence the investing choices of investors at Chinese stock markets. Four behavioral aspects of the herding factor are all connected to imitating the activities of other investors. Price variations, market knowledge, and previous stock movement are the three elements that make up the market factor. The prospect factor consists of four components: mental accounting (with two sub-variables), mental accounting (with loss aversion and regret aversion), and mental accounting. Two components make up the heuristic variables: overconfidence-gambler’s fallacy and anchoring-ability bias. In contrast to the anchoring-ability bias component, which consists of two variables: ability bias and anchoring, the overconfidence-gambler’s fallacy factor consists of two variables: overconfidence and gambler’s fallacy. The decisions that investors make are affected by all of these variables taken together.

The results of the investigation show that Hypothesis H1 is largely supported. Prospect, herding, and heuristic (containing two sub-elements) are the behavioral factors that have the most moderate influence on individual investors’ decisions. Herding speed and the gambler’s fallacy are two elements that have less of an effect on the decisions made by investors. It’s interesting to note that when making investing decisions, three market factors—price movements, market knowledge, and historical stock trends—as well as one prospect component element—mental accounting—come into play. Only three variables—herding, prospect (which includes loss aversion, regret aversion, and mental accounting), and heuristic (which includes overconfidence and gambler’s fallacy)—have been found to significantly affect investing success. Among these, heuristic behaviors instead of herding behaviors have a more favorable impact on the outcome of investments. The favorable influence of heuristic behaviors is bigger than that of the other two components. Conversely, prospect behaviors yield a negative impact on investment performance. These findings diverge from Hypothesis H2, which proposed that all behavioral factors would positively impact investment performance.

The findings underscore that a certain level of overconfidence exerts a positive effect on investment enactment. As a result, single investors should maintain a measured degree of overconfidence to effectively apply their expertise and knowledge in specific situations, thus enhancing investment outcomes. Particularly in times of uncertainty, overconfidence can prove beneficial by empowering investors to tackle challenging tasks and aiding them in forecasting future trends. In addition to overconfidence, herding is also observed to have a favorable impact on investment performance. Therefore, single investors are advised to establish partnerships or alliances with competent investment peers, leveraging their insights as valuable references for making informed decisions. Creating platforms for mutual support and information-sharing within forums can contribute to accessing reliable stock market information. Prospect considerations, on the other hand, have a detrimental effect on investment performance, according to the data. In light of their possible negative impact on investing decision-making, investors should proceed cautiously when dealing with loss aversion, regret aversion, and mental accounting.

The recommendations for investors include being diligent in their investment decisions, while also avoiding excessive fixation on prior losses for subsequent investment choices. Striking this balance is crucial to prevent missed investment opportunities, mitigate potential negative psychological impacts, and ultimately improve investment performance. Given certain limitations, the current research concentrates solely on the actions of individual stockholders in the Chinese stock markets. To gain a comprehensive understanding of the Chinese stock market landscape, further research should encompass the behaviors of institutional investors. This broader perspective would contribute to a more holistic and well-rounded assessment of the market dynamics. The study has a limited sample size due to resource constraints, potentially failing to represent the broader diversity of Chinese investors. Findings of this study are not applicable in general due to regional, cultural, or economic variations within China. Moreover, the study used convenient sampling so findings of the study cannot be generalized. Reliance on self-reported data or surveys could introduce response bias or inaccuracies due to subjective perceptions of participants. Market conditions and behavioral trends are dynamic. The study captures a snapshot of behavior at a specific time, which might not reflect long-term patterns or changes in market dynamics. Moreover, the study did not account for external factors such as regulatory changes, geopolitical events, or economic fluctuations, which can significantly influence investor behavior. Focusing on specific behavioral aspects might overlook other influential factors like socioeconomic status, education, or personal experiences that also shape investment decisions. Addressing these limitations often strengthens the credibility and applicability of such studies, allowing for a more comprehensive understanding of the behavioral dynamics influencing investment decisions among Chinese investors.

## Supporting information

S1 Data (XLSX)
